RETRACTED

# Mechanisms of Hybrid Oligomer Formation in the Pathogenesis of Combined Alzheimer's and Parkinson's Diseases

**DOI:** 10.1371/journal.pone.0003135

**Published:** 2008-09-04

**Authors:** Igor F. Tsigelny, Leslie Crews, Paula Desplats, Gideon M. Shaked, Yuriy Sharikov, Hideya Mizuno, Brian Spencer, Edward Rockenstein, Margarita Trejo, Oleksandr Platoshyn, Jason X.-J. Yuan, Eliezer Masliah

**Affiliations:** 1 Department of Chemistry and Biochemistry, University of California San Diego, La Jolla, California, United States of America; 2 Department of Neurosciences, University of California San Diego, La Jolla, California, United States of America; 3 Department of Pathology, University of California San Diego, La Jolla, California, United States of America; 4 Department of Medicine, University of California San Diego, La Jolla, California, United States of America; 5 San Diego Super Computer Center, University of California San Diego, La Jolla, California, United States of America; National Institutes of Health, United States of America

## Abstract

**Background:**

Misfolding and pathological aggregation of neuronal proteins has been proposed to play a critical role in the pathogenesis of neurodegenerative disorders. Alzheimer's disease (AD) and Parkinson's disease (PD) are frequent neurodegenerative diseases of the aging population. While progressive accumulation of amyloid β protein (Aβ) oligomers has been identified as one of the central toxic events in AD, accumulation of α-synuclein (α-syn) resulting in the formation of oligomers and protofibrils has been linked to PD and Lewy body Disease (LBD). We have recently shown that Aβ promotes α-syn aggregation and toxic conversion *in vivo*, suggesting that abnormal interactions between misfolded proteins might contribute to disease pathogenesis. However the molecular characteristics and consequences of these interactions are not completely clear.

**Methodology/Principal Findings:**

In order to understand the molecular mechanisms involved in potential Aβ/α-syn interactions, immunoblot, molecular modeling, and *in vitro* studies with α-syn and Aβ were performed. We showed *in vivo* in the brains of patients with AD/PD and in transgenic mice, Aβ and α-synuclein co-immunoprecipitate and form complexes. Molecular modeling and simulations showed that Aβ binds α-syn monomers, homodimers, and trimers, forming hybrid ring-like pentamers. Interactions occurred between the N-terminus of Aβ and the N-terminus and C-terminus of α-syn. Interacting α-syn and Aβ dimers that dock on the membrane incorporated additional α-syn molecules, leading to the formation of more stable pentamers and hexamers that adopt a ring-like structure. Consistent with the simulations, under *in vitro* cell-free conditions, Aβ interacted with α-syn, forming hybrid pore-like oligomers. Moreover, cells expressing α-syn and treated with Aβ displayed increased current amplitudes and calcium influx consistent with the formation of cation channels.

RETRACTED

**Conclusion/Significance:**

These results support the contention that Aβ directly interacts with α-syn and stabilized the formation of hybrid nanopores that alter neuronal activity and might contribute to the mechanisms of neurodegeneration in AD and PD. The broader implications of such hybrid interactions might be important to the pathogenesis of other disorders of protein misfolding.

## Introduction

Misfolding and pathological aggregation of neuronal proteins has been proposed to play a critical role in the pathogenesis of neurodegenerative disorders [1]–[3]. Dimeric forms of misfolded proteins can form propagating oligomers [4]–[6], and aggregates adopting a globular or protofibrillar shape might represent some of the toxic species [7]. However there might be a wide heterogeneity in the size and conformation of the toxic oligomers [6], 8.

Alzheimer's disease (AD) and Parkinson's disease (PD) are the leading neurodegenerative disorders in the aging population resulting in dementia and movement disorders. Over 5 million people live with these devastating neurological conditions in the US and it is estimated that this country alone will see a 50% annual increase of AD and PD by the year 2025 [9]. In AD, amyloid-β protein (Aβ)—generated from the proteolytic cleavage of the amyloid precursor protein (APP)—accumulates in the intracellular [10]–[13] and in the extracellular space, leading to the formation of plaques [14]. In PD, intracellular accumulation and fibrillization of α-synuclein (α-syn)—an abundant synaptic terminal protein [15]—results in the formation of characteristic inclusions denominated Lewy bodies (LBs) [16]–[21].

Previous studies suggest that in disorders of protein misfolding, the accumulation of oligomers and protofibrils rather than fibrils might be the neurotoxic species [22]. While progressive accumulation of Aβ oligomers has been identified as one of the central toxic events in AD leading to synaptic dysfunction [3], [6], [8], accumulation of α-syn resulting in the formation of oligomers and protofibrils that disrupt membrane and mitochondrial activity has been linked to PD [23]–[25].

The mechanisms through which Aβ and α-syn aggregates might lead to neurodegeneration are the subject of intense investigation. Various lines of evidence support the contention that abnormal aggregates arise from a partially folded intermediate precursor that contains hydrophobic patches. It has been proposed that the intermediate oligomers form annular protofibrils and pore-like structures [1], [26]–[28] that might allow the abnormal flow of ions such as Ca^2+^ [29], [30]. Most studies have been focused on studying the formation of toxic oligomeric species derived from homologous monomers, however it is possible that heterologous molecules might also interact to form toxic hybrid oligomers.

RETRACTED

For example, we have previously shown that Aβ promotes α-syn aggregation and toxicity *in vivo* [31], and that Aβ and α-syn might directly interact *in vitro* [32]. This is of interest because several studies have now confirmed that the pathology of AD and PD overlap in a heterogeneous group of conditions denominated jointly as Lewy body disease (LBD) [19], [33]–[37]. While in patients with dementia with Lewy bodies (DLB) the clinical presentation is of dementia followed by parkinsonism, in patients with Parkinson's disease dementia (PDD) the initial signs are of parkinsonism followed by dementia [34], [38]–[40].

Although these studies suggest that interactions between α-syn and Aβ are involved in the pathogenesis of LBD, the molecular characteristics and consequences of these interactions are not completely clear. For this purpose, a dynamic model investigating the early steps of Aβ and α-syn co-aggregation was developed using computer simulations that include the molecular dynamics (MD) process of protein-protein and protein-membrane docking with measurements of energies of interaction. These studies were supported by electron microscopy, *in vitro*, and *in vivo* studies in transgenic (tg) mice to further characterize the nature of Aβ and α-syn interactions.

Our studies suggest that Aβ and α-syn interact *in vivo* [31] and that at early stages the N-terminal region of Aβ monomers and dimers interact with the N and C-terminus of α-syn, leading to the formation of pentamers and hexamers with a ring-like structure [4]. These ring-like aggregates are more stable compared to those lacking Aβ and might correspond to non-selective cation channels [4]. Thus, better understanding of the steps involved in α-syn aggregation and the role that Aβ plays in this process is important in order to develop intervention strategies that might prevent or reverse Aβ-mediated α-syn oligomerization and toxic conversion.

## Results

### α-Syn and Aβ directly interact in the brains of patients with LBD and in APP/α-syn tg mice

Previous studies have shown that Aβ plays a key role in promoting α-syn aggregation [31], [32], however it is unclear to what extent both of these molecules interact *in vivo*. For this purpose, immunoblot analysis was performed with brain samples from cases with LBD and APP/α-syn tg mice. Compared to non-demented controls and AD cases, in the membrane fractions of the LBD brain homogenates there was extensive accumulation of α-syn oligomers including dimers, trimers, pentamers and higher-order aggregates (**Figure 1A,B**). Similarly, in the APP/α-syn double tg animals, which produce high levels of Aβ, there was a significant increase in the levels of α-syn oligomers compared to single tg and non-tg controls (**Figure 1D,E**).

RETRACTED

**Figure 1:** Immunoblot and co-immunoprecipitation analysis of aggregated α-syn in brains of LBD cases and tg mice. (A, B) Representative western blot (A) and semi-quantitative analysis (B) of levels of α-syn dimers and oligomers in membrane fractions from the frontal cortex of age-matched non-demented control, AD and LBD brains. In cases with LBD there was a significant increase in the levels of α-syn dimers and oligomers when compared to controls. (C) Immunoprecipitation of homogenates from control, LBD and AD cases with monoclonal antibodies against Aβ (upper panel) or α-syn (lower panel). Immunoblots were probed with monoclonal antibodies against α-syn (upper panel) or Aβ (lower panel). Aβ and α-syn pure proteins were included on the immunoblots as positive controls (first and second lanes). (D, E) Representative western blot (D) and semi-quantitative analysis (E) of levels of α-syn dimers and oligomers in the membrane fractions from nontg, APP tg, α-syn tg, and APP/α-syn double tg brains. In APP/α-syn tg mice there was a significant increase in the levels of α-syn dimers and oligomers when compared to nontg or single tg animals. (F) Immunoprecipitation of brain homogenates from nontg, APP tg, α-syn tg, and APP/α-syn double tg animals with monoclonal antibodies against Aβ (upper panel) or α-syn (lower panel). Immunoblots were probed with monoclonal antibodies against α-syn (upper panel) or Aβ (lower panel). Bar graphs represent the mean of n = 4 cases per group. *P<0.05 compared to control human brains or nontg mouse brains (by one-way ANOVA with post-hoc Tukey-Kramer test).

To further investigate whether Aβ and α-syn might interact *in vivo*, co-IP studies were performed. When samples from human brains were immunoprecipitated with an antibody against Aβ and then analyzed by western blot with an antibody against α-syn, the strongest interaction was observed in the LBD cases and to a lesser extent in the AD samples but no interaction was detected in the non-demented controls (**Figure 1C**, upper panel). Moreover, when the brain samples were immunoprecipitated with an antibody against α-syn and then analyzed by western blot with an antibody against Aβ, a strong band was detected in the LBD cases followed by the AD cases, but not in the control samples (**Figure 1C**, lower panel). Similarly, when brains from the tg mice were immunoprecipated with an antibody against Aβ and then analyzed by western blot with an antibody against α-syn, the strongest interaction was observed in the in the APP/α-syn tg samples but not in the single tg mice or in the nontg controls (**Figure 1F**, upper panel). Moreover, immunoprecipitation of the mouse brain samples with an antibody against α-syn, followed by immunoblot analysis with an anti-Aβ antibody showed a strong interaction in the APP/α-syn tg but not in the single tg mice (**Figure 1F**, lower panel).

RETRACTED

### Molecular dynamics studies show that Aβ and α-syn form hybrid ring-like structures

To better understand the molecular interactions between Aβ and α-syn that lead to aggregation, we first investigated using molecular dynamics techniques the conformational changes that Aβ and α-syn undergo over time when docked to a membrane. Simulation of α-syn was performed based on the micelle-bound structure of α-syn as resolved by NMR, presuming that a molecule in the conformation formed in contact with the lipid surface was disconnected and surrounded by water molecules. These simulations have been previously described [4]. Simulation of Aβ was conducted using the mostly helical existing NMR structure of the Aβ_1–42_ peptide. The mostly helical structure of Aβ is divided into two regions (termed helix-N and helix-C) connected by a short linker (**Figure S1**). In our baseline model, the two curved helical domains formed an angle of 55° that decreased to around 34° during the first 0.5 ns of the simulation, and then increased to 52°–55° during 1.0–1.5 ns of simulation. At 2 ns the angle was at 37°, at 2.5 ns it was at 28°, and at 3 ns the angle increased to 46°. During the simulation (**Figure S1**), the linker loop between the two helical domains became larger with only two of the initial five turns of the helix remaining after 3 ns of simulation.

Further analysis consisted of determining changes in the secondary structure of Aβ over time. After 500 ps of simulation, a coiled region appeared, interrupting the C-terminal α-helix around amino acid (aa) residue 32. Beginning at 800 ps, turns appeared in the C-terminal α-helical structure around aa 27, then after 1 ns this entire region was transformed into an unstructured loop. The π-helix transformation of the α-helical structure increased consistently over time (**Figure S2**).

Since previous studies have suggested that the assembly of α-syn and Aβ oligomers might involve interactions with the membrane [26], we conducted docking of α-syn (4 ns) and Aβ (2 ns) conformers on a 1-palmitoyl-2-oleoyl-sn-glycero-3-phosphocholine (POPC) membrane with a grid cell of 1Å. Based on the MD results, studies of the interactions between Aβ and α-syn were performed by docking the structure of the 2 ns Aβ conformer to the 4 ns α-syn dimers (**Figure 2A**) and trimers. This study showed that the Aβ conformers formed complexes with the α-syn dimers and trimers and had the capability of docking on the membrane (**Figure 2B**). Most of the interactions predicted by this model occurred between the N-terminus of Aβ with the N-terminus of the α-syn molecules, however interactions with the C-terminus of α-syn were also identified (**Figure 2C,D**). The interactions of the Aβ conformer (2 ns) in the complex were divided into three groups reflecting the individual contacts of the Aβ molecule with each of the α-syn molecules in the complex (**Figure 2C**). For the first group, the negatively-charged GLU3 of Aβ interacts with the positively-charged LYS6 of the second α-syn molecule (α-syn2), and GLN15 of Aβ most probably creates an H-bond with LYS97 in the middle region of α-syn2 (**Table 1** and **Figure 2D**). For the second group, the Aβ conformer also largely interacts with the N-terminal part of the first α-syn conformer (α-syn1). Here, LEU17 of Aβ contacts LYS32 of α-syn1, PHE19 of Aβ creates hydrophobic contacts with VAL3 and PHE4 of α-syn1, ILE31 of Aβ contacts THR22 of α-syn1; and ALA42 of Aβ contacts THR33 of α-syn1 (**Table 1** and **Figure 2D**). Finally, for the third group, the Aβ conformer might also contact the third α-syn molecule part of the complex (α-syn3) creating possible electrostatic interactions between the LYS5 of Aβ and GLU123 of a third α-syn molecule. The MD simulations demonstrated that over time, these hydrophobic and electrostatic interactions were stable as reflected by the distance between the aa residues, which ranged from 2.8 to 6.8 Å (**Table 1**). Further molecular simulations showed that docking of the Aβ molecule to the α-syn dimer or trimer stabilized the complex and facilitated the docking of additional α-syn monomers resulting in the formation of pentamers and hexamers of α-syn arranged in a ring-like conformation (**Figure 2E**).

RETRACTED

**Figure 2:** Molecular dynamics studies of the interactions of one Aβ monomer with membrane-docked α-syn multimers. (A) Diagrammatic representation of the complex formed between the 2 ns Aβ conformer and the 4 ns α-syn dimer, composed of two molecules of α-syn (α-syn1 and α-syn2). (B) Molecular modeling of the Aβ monomer/α-syn dimer complex docked to the membrane. (C) Diagrammatic representation of predicted interactions between the Aβ monomer and the two α-syn molecules occur primarily between the N-terminus of Aβ and the N-terminus of the α-syn molecules (circled regions). (D) Specific residues involved in interactions between the Aβ monomer and the two α-syn molecules. (E) Docked complex of Aβ and the α-syn dimer or higher-order oligomers (trimer, pentamer) form a ring-like structure on the membrane.

**Table 1:** Aβ contact points with α-syn dimer during MD simulations.

Contact			0 ns	0.1 ns	0.5 ns	1.0 ns	Interaction
Aβ residue	α-syn1 residue	α-syn2 residue					
GLU3*		LYS6*	6.2	6.5	6.0	2.8	Electrostatic
PHE4*		ILE88*			3.9	3.6	Hydrophobic
ARG5		ILE88			4.2	6.5	Hydrophobic
ASP7		THR92			2.8	6.9	Hydrophobic
GLU11*		LYS97*		2.8	2.8	4.8	Electrostatic
VAL12*		LYS97*		4.7	4.2	4.8	Hydrophobic
VAL12*		VAL95*	3.6		6.1	4.7	Hydrophobic
VAL12*		ALA91*		3.8	4.1		Hydrophobic
HIS13	LYS32			4.2	3.6	3.7	Hbond
GLN15		LYS97	4.6	2.8			Hbond
GLN15		GLU105		5.7	6.5	6.5	Possible Hbond
LYS16*		ASP98*	4.7	2.8	2.8	2.8	Electrostatic
LYS16*	GLU28*			5.5			Electrostatic
LEU17	LYS32		4.8	4.0	5.7	6.4	Hydrophobic
PHE19	PHE4		4.7			4.6	Hydrophobic
PHE19	VAL3		5.4	4.0			Hydrophobic
ILE31	GLY25			5.3	4.4	6.3	Hydrophobic
ILE31	ALA29			5.4			Hydrophobic
ILE31	THR22		6.8				Hydrophobic
ILE31	LYS21			5.6	6.0		Hydrophobic
ILE32	VAL26		6.8		4.7	4.9	Hydrophobic
ILE32	THR22				4.1	4.0	Hydrophobic
LEU34	GLU28			3.8	4.1	4.4	Hydrophobic
LEU34	ALA29		3.8	4.4	4.5	4.1	Hydrophobic
GLU37	ALA29			6.2	4.5	4.3	Hydrophobic
GLU38	ALA29			4.4			Hydrophobic
ALA42	THR33		3.8				Hydrophobic

* Indicates residues located at the points predicted to be critical for stabilization of the Aβ-α-syn complexes on the membrane. These resides of Aβ were mutated for additional analysis of Aβ-α-syn interactions.

### Structural organization and energy of interaction of the hybrid Aβ and α-syn oligomers on the membrane

Since previous studies have suggested that the assembly of α-syn and Aβ oligomers might involve interactions with the membrane [26], [41], [42], we conducted docking of α-syn (4 ns) and Aβ (2 ns) conformers on a POPC membrane with a grid cell of 1Å, including the membrane in calculations. First, the α-syn molecules were docked to the membrane to determine the most favorable energy of interaction for the dimers, trimers and higher-order oligomers. Then, to each of the α-syn oligomers, an Aβ molecule (2 ns conformer) was docked, selecting the complexes with the most favorable (lowest) energy of interaction (**Figure 3A,B**). These simulations showed that Aβ increased the stability of the oligomers and facilitated further docking of other α-syn molecules to form pentamers and hexamers on the membrane (**Figure 3A,B**). The α-syn complexes that included Aβ displayed higher stability on the membrane and lower electrostatic energy of interaction when compared to multimers containing only α-syn (**Figure 3B**). Both Aβ monomers and dimers increased the stability of the α-syn complexes, with lower electrostatic energy of interaction of α-syn with the α-syn–Aβ monomer and α-syn–Aβ dimer complexes than with the single α-syn molecule (10–15% higher) (**Figure 3B** and **Figure S3**). The hybrid α-syn-Aβ multimers formed ring-like structures that became embedded in the simulated membrane (**Figure 3C,D**) after relatively short (350 ps) MD simulations of the membrane-proteins complex. During extended simulation times, the α-syn pentamer embedded progressively further into the membrane, reaching a depth of 1.6Å in the membrane by 800 ps (**Figure 3C,D**). Space-filled modeling also demonstrated that the complex containing Aβ and the α-syn pentamer embedded into the membrane over time (**Figure 3E,F**).

RETRACTED

**Figure 3:** Modeling and energies of interaction between Aβ and α-syn oligomers docked on the membrane. (A) Conformation of lowest-energy complex between α-syn pentamer and 2 ns Aβ conformer on the membrane. (B) Calculated values for the most favorable energies of interaction between one Aβ monomer and an α-syn monomer, dimer, trimer, tetramer or pentamer. Compared to α-syn homomeric species composed of the same number of α-syn molecules, hybrid Aβ/α-syn multimers were more stable and had more favorable (lower) electrostatic energies of interaction. (C, D) Hybrid Aβ/α-syn multimers formed ring-like structures that embedded in the membrane after 350–800 ps of simulation. (E) Space-filled model of Aβ (orange)/α-syn (gray) multimer embedded in the membrane (green) at a depth of 1.6Å after 800 ps of MD simulation. (F) Space-filled model of Aβ (orange)/α-syn (gray) multimer showing the depth of 1.6Å (purple) that the complex embedded into the membrane (POPC) after 800 ps of MD simulation. (G) Space-filled model of Aβ (green) and α-syn (red) monomer initially situated on opposite sides of the POPC membrane showing penetration of the Aβ and α-syn molecules into the membrane and interaction between the two after 2.3 ns of MD simulation.

To further investigate the potential interactions between α-syn and Aβ when the two molecules are located on the opposite sides of a membrane, we performed additional MD simulations where the 2 ns conformer of Aβ was docked on one side of the membrane, while the 4.5 ns conformer of the α-syn monomer was docked on the other side of the membrane. During the initial stage of the MD (at 1.0 ns), Aβ was in contact with the membrane at aa residues 20–33 and was embedded into to the membrane at a depth of 3Å (**Figure 3G**). In this orientation, residues 20–33 exhibit a “membranephilic” combination of hydrophobic and charged residues. The hydrophobic residues in this region interacted with the membrane by penetration into the hydrophobic parts of the lipids. During MD simulations, Aβ changed its overall orientation so that the longer N-terminal α-helix becomes more perpendicular to the membrane. During the penetration time (2.3 ns) the C-terminal α-helix of Aβ transformed to a π-helix (**Figure 3G**), with residues 29–34 forming the tip of the penetrating peptide. After 2.3 ns of MD simulation, the N-terminal region of α-syn also penetrated the membrane at a depth of 1.6Å where the two molecules came into contact with each other. It worth noting that residues GLY29, ALA30, ILE31, ILE32, GLY33, and LEU34 created a defined “hydrophobic frontal tip for penetration” as these residues can better interact with the hydrophobic parts of the lipid bilayer. Taken together, these simulation studies support the possibility that even if α-syn and Aβ might be on opposite sides of a membrane, because of their helical structures and lipid interactions they might be able to penetrate and interact at an intermediate membrane point.

RETRACTED

### The impact of Aβ on conformational stability of the α-syn initial dimer and its docking to the membrane

Recent studies have shown that during the aggregation of α-syn, formation of essentially static dimeric species is the critical first step of the aggregation process [43], and α-syn dimers are formed before other higher-order oligomers [44]. Furthermore, under certain pathological conditions, dimer formation is the rate-limiting step in α-syn aggregation [45]. Additional evidence shows that during the early phase of α-syn aggregation, a high-affinity lipid binding intermediate is formed [46], and dimers preferentially bind lipid membranes [42]. Moreover, a previous study showed that in a cell culture model, α-syn forms small oligomers, primarily dimers and trimers, that preferentially associate with cell membranes [47]. In support of these results, we have previously shown that the “initial” α-syn dimer that supports further aggregation is docked on the membrane in a head-to-head conformation [4]. This dimer can serve as the core for the formation of pentameric and hexameric oligomers with a ring-like organization. In the previous section it was shown that Aβ can bind to this initial α-syn dimer with favorable interaction energies (**Figure 3B**). Such electrostatic and van der Waals energy calculations are useful for defining the proper docking position, but these are not sufficient to evaluate the possible impact of such docking to the configuration changes of the α-syn dimer in the membrane over time. To answer this question, two sets of MD calculations in the membrane were conducted. The first was performed with the initial α-syn dimer alone, and the second with the same complex that included the 2 ns conformer of Aβ. The simulations showed that after 0.8 ns the N-terminal helices of the α-syn dimer changed their conformation and compromised the docking plane of α-syn to the membrane surface (**Figure 4A,B**). As a parameter that might represent such conformational changes, the angle between the C-alpha atoms of the residues VAL66 (α-syn1), LYS45 (α-syn1), VAL37 (α-syn2) was measured to estimate the possible surface of the protein's membrane contact plane (**Figure 4A,B,E,F**). Based on the calculations for the electrostatic energy of interactions, an angle of less than 80° allowed stable docking of the α-syn dimer to the membrane. In contrast, when the angle was greater than 80°, docking of the α-syn dimer over the time course of the MD simulations was less likely. For the α-syn dimer (without Aβ), this angle remained close to 80° for up to 0.5–0.8 ns (**Figure 4A,E,F**), however after this time the angle increased, compromising the docking of the α-syn dimer to the membrane (**Figure 4B,F**). In contrast, when Aβ was docked to the initial α-syn dimer, this angle remained within 60° to 80°, stabilizing the α-syn dimer and allowing the docking of the complex to the membrane over a longer period of time (**Figure 4C–F**).

RETRACTED

**Figure 4:** Molecular dynamics of conformational changes of membrane-associated α-syn in the presence of one Aβ monomer. (A) Initial conformation of α-syn dimer on the membrane without Aβ. (B) 0.8 ns conformation of α-syn dimer on the membrane without Aβ. (C) Initial conformation of α-syn dimer on the membrane with Aβ monomer. (D) When complexed with the Aβ monomer, after 0.8 ns the conformation of the α-syn dimer on the membrane is drawn closer to the membrane, and the α-syn molecules make more contact points with the membrane surface than the α-syn dimer alone. (E) Comparison of the two complexes at 0.8 ns demonstrating the angle measured between the C-alpha atoms of the residues VAL66 (α-syn1), LYS45 (α-syn1), VAL37 (α-syn2). The complex without Aβ had an angle of <80° (upper), while the complex with Aβ had an angle of >80° (lower) and was more stable on the membrane. (F) Changes in angle measurements in the complexes over time without Aβ or in the presence of wild-type or mutated full-length Aβ. In the mutated Aβ peptide, positively-charged residues were substituted for negative ones and hydrophobic residues for hydrophilic ones (PHE4SER, GLU11ARG, VAL12SER, LYS16ASP).

RETRACTED

Next, to determine which residues of Aβ were the most critical to the stabilization of the α-syn dimer during the course of the MD studies, additional simulations were performed with mutated forms of the full-length Aβ molecule. Inter-molecular interactions that remained stable over the course of the MD simulations were those between amino acids that formed electrostatic contacts between residues with opposite charges such as GLU3 (Aβ) and LYS6 (α-syn2), and LYS16 (Aβ) and ASP98 (α-syn2) (**Table 1**). Other strong but less stable contacts were the electrostatic interactions between GLU11 (Aβ) and LYS97 (α-syn2), and hydrophobic interactions between VAL12 (Aβ) and VAL95 (α-syn2), and PHE19 (Aβ) and PHE4 (α-syn1) (**Table 1**), where α-syn1 is to the left (depicted in magenta) and α-syn2 is to the right (depicted in brown) in the dimer (**Figure 2A**). Remarkably, when the MD simulations were performed with the initial α-syn dimer and a mutated Aβ molecule (PHE4SER, GLU11ARG, VAL12SER, LYS16ASP), the stability of the dimer docking over time was compromised, with the angle increasing to greater than 80° after 0.7 ns of the MD simulation (**Figure 4F**).

### Aβ and α-syn form hybrid ring-like structures in an *in vitro* cell-free system

In the brains of patients with AD and LBD both monomeric and oligomeric forms of α-syn and Aβ may be present, however it is unclear if the interactions leading to aggregation are only between monomers or also between monomers and oligomers. The MD simulations and the electrostatic energy calculations suggest that in addition to the interactions between monomers and dimers, interactions between oligomers are also possible. To investigate this possibility, aggregated or freshly-solubilized Aβ and α-syn were co-incubated and analyzed by immunoblot. Consistent with our previous studies [31], freshly-solubilized Aβ_1–42_ promotes the aggregation of soluble α-syn in an *in vitro* cell-free system in a dose and time-dependent manner (**Figure S4**). In order to investigate the conformational change of these proteins, immunoblot analyses were performed with aggregated and freshly-solubilized Aβ and α-syn co-incubated under comparable conditions (**Figure 5A,B**). This study showed that solubilized Aβ induced aggregation of α-syn into tetramers and higher-order oligomers with changes in electrical charge, suggesting that Aβ induced conformational change in α-syn (**Figure 5A**). Pre-aggregated Aβ promoted the formation of stable dimers and trimers of α-syn and, to a lesser extent, higher-order aggregates (**Figure 5A**). By immunoblot, freshly-solubilized Aβ appeared mostly as a single band at a molecular weight of 4 kDa, and aggregated as a series of immunoreactive bands consistent by with the expected molecular weight of dimers, trimers and tetramers (**Figure 5B**). Next, *in vitro* binding assays were performed to verify if α-syn and Aβ directly interact in the *in vitro* cell-free system. For this purpose, the α-syn and Aβ protein complexes were immunoprecipitated with a polyclonal anti-α-syn antibody, followed by immunoblot analysis with a monoclonal anti-α-syn antibody or anti-Aβ antibody. Western blot analysis demonstrated that α-syn in the mixture was precipitated by the antibody (**Figure 5C**). Co-immunoprecipitated Aβ was detected in the presence of α-syn but not in the absence of α-syn (**Figure 5D**), supporting the notion that α-syn and Aβ directly interact.

RETRACTED

**Figure 5:** Interactions between Aβ and α-syn in an *in vitro* cell-free aggregation model. Freshly-solubilized or pre-aggregated Aβ_1–42_ was incubated at concentrations of 10 or 20 µM (as indicated) with freshly-solubilized recombinant α-syn and samples were analyzed by immunoblot or co-immunoprecipitation. (A) Increased levels of α-syn high-molecular weight forms aggregates in the presence of freshly-solubilized or pre-aggregated Aβ, as shown by immunoblot analysis with a polyclonal antibody against α-syn. (B) Formation of Aβ multimers after incubation under aggregating conditions. (C, D) *In vitro* binding assay for Aβ and α-syn. Immunoprecipitation of cell-free aggregated samples was performed using a polyclonal antibody against α-syn. Immunoblots were probed with monoclonal antibodies against α-syn (C) or Aβ (D). Aβ was only detected in samples that were incubated with α-syn, and in cases where no recombinant protein was included (negative control), no immunoreactivity was detected with either antibody. (E, F) Samples containing freshly-solubilized α-syn were incubated with the following peptides: an 18-mer N-terminal fragment of Aβ containing mutations at the residues determined to be critical for interaction with α-syn (Aβ mut), an 18-mer N-terminal fragment of Aβ of the wild-type sequence (Aβ wt), or full-length Aβ_1–42_ peptide (Aβ 1–42) and analyzed by immunoblot with an antibody against α-syn. Incubation with the Aβ mut resulted in lower levels of the dodecamer form of α-syn. The sequence of the wt and mut Aβ peptides (18-mers) used for these experiments are shown in panel e. Arrows indicate mutated residues.

To determine if the Aβ residues identified by the simulations as critical to stabilizing α-syn dimers on the membrane and promoting further aggregation of α-syn, an additional experiment was performed with a mutated N-terminal fragment of Aβ (18 aa in length). For this purpose, recombinant α-syn was incubated with a mutated Aβ peptide where positively-charged residues were substituted for negative ones and hydrophobic residues for hydrophilic ones (PHE4SER, GLU11ARG, VAL12SER, LYS16ASP). Immunoblot analysis confirmed that while the peptide corresponding to the wild type N-terminal 18 aa sequence of Aβ_1–42_ promoted α-syn aggregation like the full-length Aβ_1–42_ peptide, the mutated version of the Aβ peptide was less effective (**Figure 5E,F**).

RETRACTED

### Aβ enhances the formation of α-syn ring-like structures and increases ion conductance alterations

Previous studies have shown *in vitro* that Aβ [48] and α-syn aggregates can independently form oligomers with a ring-like morphology [25], [49]. However the ultrastructural characteristics of the hybrid Aβ and α-syn multimers are unclear. Consistent with the MD simulations and the immunoblot analysis, electron microscopy studies showed that compared to the vehicle control (**Figure 6A**), when incubated separately for 6 hrs, Aβ and α-syn generated ill-defined globular structures ranging in size between 5 to 10 nm (**Figure 6B,C**). In contrast, at 6 hrs the mixture between Aβ and α-syn resulted in well-defined ring-like structures measuring 9–15 nm with a central channel of approximately 3–5 nm (**Figure 6D**). The mixture of Aβ and α-syn showed increased numbers of ring-like structures after 6 hrs (**Figure 6E**). At longer periods of incubation, Aβ and α-syn alone, and the mixture formed fibrils of approximately 11 nm in diameter that increased in number in the samples containing a mixture of Aβ and α-syn (**Figure 6F–I**).

**Figure 6:** Electron microscopy analysis of hybrid oligomers and fibrils of Aβ and α-syn. *In vitro* cell-free preparations of vehicle, Aβ alone, α-syn alone, or Aβ and α-syn were incubated for 6 hrs or 48 hrs and prepared for electron microscopy analysis. (A–D) After 6 hrs of incubation, compared to vehicle alone (A), Aβ (B) and α-syn (C) alone formed globular structures of 5–10 nm in diameter, while incubation of Aβ and α-syn together (D) resulted in the formation of larger, well-defined ring-like structures with a central channel. (E) Analysis of numbers of ring-like structures formed after 6 hrs incubation. (F–I) After 48 hrs of incubation, compared to vehicle alone (F), Aβ (G) and α-syn (H) alone or in combination (I) formed fibrils of about 11 nm in diameter. (J–M) After 6 hrs incubation in the presence of lipid monolayers, compared to vehicle alone (J), Aβ (K) and α-syn (L) alone formed globular structures of 5–8 nm in diameter, while incubation of Aβ and α-syn together (M) resulted in enhanced formation of larger, well-defined, ring-like structures. Scale bar, 10 nm (A–D, J–M); 100 nm (F–I).

RETRACTED

Since MD simulations were performed in a membrane-based model, in order to determine if similar interactions occur between Aβ and α-syn in the presence of organic lipids, ultrastructural studies were performed on cell-free protein preparations that were incubated with lipid monolayers for 6 hrs. Electron microscopy analysis confirmed that in the presence of lipids, both Aβ (**Figure 6K**) and α-syn (**Figure 6L**) alone form ring-like structures measuring approximately 5–8 nm in diameter compared to vehicle control (**Figure 6J**), while in the samples containing a mixture of Aβ and α-syn, this effect was enhanced (**Figure 6M**). This suggests that membrane-like lipids facilitate the formation of Aβ/α-syn hybrid ring-like structures.

Since previous studies have suggested that the α-syn ring-like structures might form pores in the membrane that could be responsible for the neurotoxic effects of α-syn oligomers [25], [26], [28], [30], we investigated whether abnormally high levels of ion currents are detected in cells over-expressing α-syn and if this process might be enhanced by Aβ. For this purpose, we recorded and compared whole-cell cation currents in human embryonic kidney (HEK) 293T cells transduced with lentiviral (lenti) vectors expressing α-syn or green fluorescent protein (GFP) as a control in the presence or absence of Aβ (**Figure 7**). Immunoblot analysis confirmed that cells expressed comparable levels of α-syn (**Figure 7A**). Double-labeling verified that in co-transduced cells, GFP was also expressed with α-syn (**Figure 7B**). The target cells (displaying green fluorescence) for electrophysiological measurements were identified by co-transduction with the lenti-GFP vector (**Figure 7B**).

**Figure 7:** Electrophysiological analysis of the cellular effects of hybrid Aβ/α-syn multimers. 293T cells were infected with lenti-α-syn and lenti-GFP and treated with Aβ and analyzed by electrophysiology. (A) Immunoblot analysis showing expression levels of α-syn and GFP in treated cultures. (B) Immunocytochemical analysis demonstrating high efficiency of infection and co-localization between α-syn and GFP. (C, D) Representative currents (C) elicited by depolarizing the cells from a holding potential of −50 mV to a series of test potentials ranging from −80 mV to +80 mV, and corresponding current voltage-relationship curves (D), in α-syn-expressing cells treated with vehicle (α-syn, n = 5), vector-transfected cells treated with Aβ (Aβ, n = 5), and α-syn-expressing cells treated with Aβ (α-syn+Aβ, n = 6).

The whole-cell cation currents were elicited by depolarizing the cells from a holding potential of −50 mV to a series of test potentials ranging from −80 mV to +80 mV in 20-mV increments. When compared to baseline conditions (i.e., cells infected with an empty vector or with lenti-GFP), the amplitude of currents was increased in cells expressing α-syn and treated with vehicle as well as in cells transduced with an empty vector and treated with Aβ (**Figure 7C,D**). Moreover, the amplitude of currents in α-syn-transduced cells treated with Aβ was much greater than that in α-syn-transduced cells treated with vehicle and in vector-transduced cells treated with Aβ (**Figure 7C,D**). The current amplitude at +80 mV was 374.6±25.5 pA in cells transduced with an empty vector (n = 10), 1467.7±152.2 pA in α-syn-expressing cells (*P*<0.001 vs. vector control), 2172.7±126.8 pA in vector cells treated with Aβ (*P*<0.001 vs. vector control; *P*<0.01 vs. α-syn-expressing cells), and 3640.3±824.6 in cells transduced with α-syn and treated with Aβ (*P*<0.001 vs. vector control; *P*<0.05 vs. α-syn-expressing cells) (**Figure 7C,D**).

RETRACTED

Recent studies have shown that the α-syn oligomers might increase the influx of calcium [30], [50]. Thus, it is possible that in our model the hybrid α-syn and Aβ complexes might also promote cellular dysfunction via abnormal influx of calcium. To investigate this possibility, levels of intracellular calcium were determined with the fluorescent calcium indicator Fluo-4. Compared to cells infected with a control lentiviral vector, the α-syn-expressing cells displayed a two-fold increase in intracellular calcium. Similar effects were observed in un-infected cells treated with Aβ. The α-syn-expressing cells treated with Aβ displayed an even greater increase in calcium levels compared to controls (**Figure S5**). Taken together, these data indicate that Aβ and α-syn form functional cation nanopores that might lead to cellular dysfunction by calcium influx.

## Discussion

Previous studies have focused on understanding the formation of toxic oligomeric species derived from homologous monomers. In the present study we show for the first time that heterogeneous proteins can form toxic hybrid oligomers. Here we demonstrate that Aβ and α-syn directly interact *in vivo* and *in vitro*. Supporting these findings, Aβ and α-syn co-immunoprecipitated in the brains of patients with LBD as well as in double APP/α-syn tg mice. Furthermore, molecular modeling studies showed that these interactions promoted the formation of highly stable ring-like oligomers composed of both Aβ and α-syn and dock in the membrane. Similarly, *in vitro* studies confirmed that both freshly-solubilized as well as aggregated Aβ and α-syn can directly interact and form hybrid ring-like structures.

RETRACTED

These findings are consistent with a previous study utilizing a different line of APP tg mice that showed that Aβ promotes the aggregation of α-syn *in vivo* and worsens the deficits in α-syn tg mice [31]. Moreover, α-syn has also been shown to accumulate in the brains of APP tg [51] and APP/presenilin-1 (PS1) double tg mice that produce large amounts of Aβ [52]. More importantly, several studies have now shown that in the brains of LBD patients, Aβ contributes to the levels and state of α-syn aggregation and LB formation [19], [32], [53]–[57]. Taken together, these studies in tg mice and human brains support the contention that Aβ and α-syn interact *in vivo* and that these interactions are of significance in the pathogenesis of the disease.

Aβ might promote α-syn aggregation by directly interacting with α-syn molecules bound to the membrane and therefore facilitating the formation of more stable oligomers. However, Aβ might promote α-syn aggregation through other pathways, including increased oxidative stress, calpain activation with C-terminal cleavage of α-syn [58], [59] and aberrant phosphorylation induced by secreted forms of Aβ. Under physiological conditions, soluble Aβ can be identified in the cytosolic fraction, in the endoplasmic reticulum and in endosomes [60], [61]. Similarly, monomeric α-syn is primarily found in the cytosolic fraction [15] and is loosely associated with synaptic vesicles [62]–[64] where it might play a role in neurotransmitter release. Moreover, monomeric α-syn can be found in lipid rafts, which is required for the synaptic localization of α-syn [62]. However, under pathological conditions, both aggregated Aβ and α-syn might associate with membranes and accumulate in caveolae [62], [64]–[71]. These specialized domains in the membrane are rich in cholesterol and sphingolipids and have been proposed to play a role in integrating signaling pathways [72]–[75]. Under pathological conditions, lipid rafts in the membrane have been postulated to play a role in oligomerization of misfolded proteins [66], [67], [76] including α-syn [62], [70], [71] and Aβ [65]–[67] and might represent a suitable site for the abnormal interactions between aggregated forms of α-syn and Aβ. In addition, these interactions might occur in other organelles such as mitochondria, multivesicular bodies and lysosomes since aggregated forms of Aβ and α-syn have been independently described in these membranous structures [23], [77]–[79]. Alternatively, given the role of lipid rafts in the synaptic localization of monomeric α-syn, it is possible that disruption of the physiological interaction of α-syn with lipid rafts may result in changes in α-syn that contribute to the pathogenesis of PD [62].

RETRACTED

Moreover, Aβ [80] and α-syn oligomers [47], [81], [82] are known to interact with membrane-like lipids and to form ring-like structures [1], [7], [41], [48], [83]. For example, in the case of α-syn, interactions with brain membranes [26] or phospholipid bilayers or vesicles that model biological membranes results in conformational modifications that facilitate oligomerization and formation of ring-like assemblies [41], [64], [84]. It is also important to note that while interaction of α-syn with biological membranes may inhibit the formation of fibrils and protofibrils [84], membrane interaction facilitates the formation of lower order oligomers because it promotes the docking of the propagating dimers [4]. In support of this, Giannakis et al recently showed that α-syn dimers preferentially bind lipid membranes, while trimers and tetramers were also detected on the lipid surface [42]. More detailed studies of the structure and organization of these aggregates have been sparse because of the difficulties in producing microcrystals of the oligomers suitable for X-ray analysis. Because of the inherent limitations in elucidating the precise structure of such transient intermediate species as oligomers, most studies have focused on *in silico* analyses [85].

The simulations and modeling in the present study suggest that anchoring of propagating α-syn complexes with Aβ to the membrane facilitates the incorporation of additional α-syn monomers, leading to the formation of trimers, tetramers, pentamers, and hexamers—the latter oligomers forming ring-like structures. The hybrid multimers of Aβ and α-syn might embed in the membrane, leading to the formation of nanopore-like structures resulting in abnormal ion conductance.

Previous studies have shown that Aβ penetrates in the membrane and aggregates to form channels that facilitate the abnormal trafficking of cations such as Ca^2+^ and K^+^ [29], [86]–[88]. Studies of α-syn aggregation by atomic force microscopy have shown that the oligomers form heterogeneous pore-like structures that might induce cell death via disruption of calcium homeostasis [49], [50]. This is in agreement with the present study showing that the hetero-multimers of Aβ and α-syn promote abnormal calcium influx. Moreover, recent studies have shown that helical α-syn forms highly conductive ion channels [89] and human neuronal cells expressing mutant α-syn have high plasma membrane ion permeability sensitive to calcium chelators [30] and that cells transduced with α-syn display significant increases in Zn^2+^-sensitive ion channel activity that might correspond to Zn^2+^-sensitive non-selective cation channels [4]. Taken together, these results support the contention that Aβ and α-syn aggregates might form functional ion-permeable channels that might play a role in the mechanisms of neurodegeneration in LBD.

RETRACTED

There is growing evidence that pathological interactions among misfolded molecules might play an important role in the formation of neurotoxic oligomers that accumulate in AD, LBD and other dementias. Remarkably, Aβ has also been shown to promote the accumulation of Tau [90], a microtubule binding protein present in the tangles in AD and fronto-temporal dementia (FTD), and the C-terminus of α-syn has been shown to interact with Tau under abnormal conditions [91]. Along these lines, our molecular dynamics studies showed that the termini of the Aβ molecule recognize specific aa in different regions of the two α-syn molecules. Interestingly, aa residues in the C-terminus of Aβ interact primarily with residues in the N-terminus of the first α-syn molecule (aa 3–33, **Table 1**), which is consistent with a previous study identifying a novel Aβ-binding domain within residues 1–56 of α-syn [92]. The N-terminus of Aβ favors interaction with residues primarily in or near the non-amyloid component (NAC) region of the second α-syn molecule (aa 88, 91, 92 and 95, **Table 1**), which is consistent with previous biochemical data [93]. The misfolded Aβ monomers and dimers might serve as a bridge across α-syn dimers and trimers, increasing the stability of the oligomers and the formation of ring-like structures in the membrane.

In conclusion, the present study showed that Aβ and α-syn interact *in vivo* in the brains of patients with LBD and in tg mice and that these interactions might result in the formation of stable hybrid ring-like oligomers in the membranes accompanied by abnormal channel activity. Therefore, developing strategies that might prevent Aβ and α-syn interactions might represent a viable target for the development of approaches for the treatment of combined AD and PD. Moreover, this study brings to light the concept of the formation of hybrid oligomers and their role in the pathogenesis of neurodegenerative disorders. Similar interactions among other heterogeneous proteins such as prion protein, huntingtin, A-Bri, and tau might be at play in other disorders of protein misfolding.

## Materials and Methods

### Molecular dynamics simulations and modeling of α-syn and Aβ

The modeling and simulations were based on the previously reported NMR structure of α-syn (PDB index 1xq8 [94]) and Aβ (PDB index 1IYT). The molecules were then minimized for 10,000 iterations of steeped descent with the Discover program (Accelrys, San Diego, CA). Molecular dynamics simulations of α-syn and Aβ molecules were conducted using periodic boundary conditions at constant pressure (1 atm) and temperature (310 K) with the water box in which the shortest distance between the protein molecule and the box walls was 30Å. The NAMD molecular dynamics program version 2.5 [95] was used with the CHARMM27 force-field parameters [96] to simulate the behavior of α-syn and Aβ molecules in water under normal conditions and the interaction of the POPC membrane with the α-syn aggregates. The temperature was maintained at 300 K by means of Langevin dynamics using a collision frequency of 1/ps. A fully flexible cell at constant pressure (1 atm) was employed using the Nosé-Hoover Langevin Piston algorithm [97], [98] as used in the NAMD software package.

RETRACTED

Initial coordinates were taken from a previously equilibrated 500 ps system. The van der Waals interactions were switched smoothly to zero over the region 10Å and electrostatic interactions were included via the smooth particle-mesh Ewald summation [99]. The impulse-based Verlet-I/r-RESPA method [100], [101] was used for multiple time-stepping: 4 fs for the long-range electrostatic forces, 2 fs for short-range nonbonded forces, and 1 fs for bonded forces. The simulation was done in four steps. Initially the system of protein and water molecules was minimized for 10,000 iterations. Then the system was heated in 0.1° increments and equilibrated for 10 ps; then the molecular dynamics simulation was conducted. Data for analysis were taken between 50 ps and 5 ns of the simulation.

### Aβ and α-syn interactions and docking to the membrane

Interactions between Aβ and α-syn monomers, dimers, and trimers, were studied using the programs Hex 4.5 [102], [103] and the docking module of Insight II (Accelrys) with a 1Å grid and cut-off distance of 20Å. Taking into account previous studies [82] showing that α-syn and Aβ aggregation occurs on the membrane, we also studied docking of molecules on a flat surface representing the plasma membrane as previously described [4]. We also simulated the behavior of pentamers formed from α-syn with Aβ on the POPC membrane. The explicit (all-atom) membrane models were utilized for simulation. Because the docking configurations of the proteins were mostly open to solution, we used a dielectric constant of 16 to calculate the electrostatic energy for α-syn and Aβ docking.

For predicting membrane-contacting surfaces of proteins we developed the program MAPAS, based on calculations of membrane-association scores for proteins and protein aggregates [104]. This program was applied to intermediate α-syn and Aβ conformers and top scoring predicted membrane attractive surfaces were used to dock the protein molecules and to subsequently calculate possible α-syn–α-syn and α-syn–Aβ docking configurations on the membrane. Low energy α-syn/α-syn propagating complexes were used in simulations of consecutive docking of the next α-syn molecules. To estimate the possible surface of the α-syn dimer contact with the membrane that changes during MD simulations we measured the angle between the C-alpha atoms of three residues: VAL66 (α-syn1), LYS45 (α-syn1), VAL37 (α-syn2) using the InsightII program (Accelrys) for each 10 ps MD conformation of the α-syn dimer.

RETRACTED

In order to investigate the dynamics of Aβ/α-syn interactions when the molecules are separated by a membrane, we also conducted MD simulations of the system containing one Aβ molecule (2 ns conformer) on one side of the membrane, and one α-syn molecule (4.5 ns conformer) on the other side of the membrane. We also conducted MD simulations of the system containing the α-syn pentamer with Aβ molecule docked to the one of the α-syn–α-syn interfaces and the POPC membrane. The pentamer of the α-syn molecules was constructed by minimal energy docking of the 4 ns conformers of α-syn (as described in our previous publication [4]). The Aβ molecule (2 ns MD conformer from the previous MD simulation of Aβ in water) has been docked to the minimal energy position in the interface between two α-syn molecules. The between two α-syn pentamer complexed with the Aβ monomer was located on the surface of the membrane with the shortest contacts between the protein docked to the membrane in the range of 3Å. The explicit (all-atom) POPC membrane model was utilized for simulation. The simulation was done in four steps. Initially the system of protein, membrane, and water molecules was minimized for 10,000 iterations. Then the system was heated in 0.1° increments and equilibrated for 500 ps; then the MD simulation was conducted using periodic boundary conditions at constant pressure (1 atm) and temperature (310 K) with the water box in which the shortest distance between the protein molecule and the box walls was 30Å. The NAMD molecular dynamics program version 2.5 [95] was used with the CHARMM27 force-field parameters [96]. The temperature was maintained at 300 K by means of Langevin dynamics using a collision frequency of 1/ps. A fully flexible cell at constant pressure (1 atm) was employed using the Nosé-Hoover Langevin Piston algorithm [97], [98] as used in the NAMD software package. The van der Waals interactions were switched smoothly to zero over the region 10Å and electrostatic interactions were included via the smooth particle-mesh Ewald summation [99]. The impulse-based Verlet-I/r-RESPA method [100], [101] was used for multiple time-stepping: 4 fs for the long-range electrostatic forces, 2 fs for short-range nonbonded forces, and 1 fs for bonded forces. Data for analysis were taken each 10 ps of the simulation.

RETRACTED

### Immunoprecipitation assays

Briefly, homogenates from human brains and transgenic mice were lysed in buffer A (20 mM Tris-HCl, pH 7.5, 150 mM NaCl, 1 mM EDTA, 1 mM NaVO4, 50 mM NaF, with protease inhibitors (Roche, Basel, Switzerland)) containing 1% Triton X-100. Immunoprecipitation assays were carried out essentially as previously described [105]. The lysates were then centrifuged for 20 min for 12,000 rpm, and the protein concentrations were determined with a BCA protein assay kit. Three hundred µg of the supernatants was incubated with 1 µg of polyclonal antibody against α-syn (Cell Signaling, Danvers, MA) overnight at 4°C, and then the immunocomplexes were adsorbed to protein A-Sepharose 4B (Amersham, Piscataway, NJ). After washing extensively with buffer A containing 1% Trion X-100, samples were heated in SDS sample buffer for 5 min and subjected to gel electrophoresis on tris-tricine gels followed by immunoblot analysis with an antibody against α-syn (Cell Signaling) or Aβ (6E10, Signet Laboratories, Dedham, MA). Also samples were immunoprecipitated with an antibody against Aβ (6E10), and run on a Bis-Tris 4–20% gel followed by immunoblot analysis with a mouse monoclonal antibody against α-syn (BD, Franklin Lakes, NJ).

### Tissue samples

A total of 12 cases (n = 4 non demented controls; n = 4 Alzheimer's Disease and n = 4 dementia with Lewy bodies- DLB) from the ADRC at UCSD were included for immunoblot analysis. All cases were carefully characterized clinically and neuropathologically and had lees than 8 hrs postmortem. The most common cause of death was bronchopneumonia and sepsis followed by renal and heart failure. The diagnosis of AD was based on the Consortium to Establish a Registry for AD (CERAD) and National Institute of Aging (NIA) criteria for diagnosis [106], [107]. The diagnosis of DLB was based on the clinical presentation of dementia and the pathological findings of Lewy bodies (LBs) detected using anti-ubiquitin and anti-α-syn antibodies as recommended by the Consortium on DLB criteria for a pathologic diagnosis of DLB [107]. In addition to the presence of LBs, the DLB cases had abundant plaques in the neocortex and limbic system but fewer tangles compared to AD cases. The DLB group belongs to a more general heterogeneous group of conditions with dementia and parkinsonism denominated Lewy body disease (LBD).

RETRACTED

For studies in animal models, brain samples from 16 mice (n = 4 nontg; n = 4 APP tg; n = 4 −α-syn tg and n = 4 APP/α-syn double tg mice were included for immunoblot analysis. For this purpose, 6-month old nontg, single (APP or α-syn tg) and double tg (APP/α-syn tg) mice were utilized. The characteristics of thy1-APPmut tg (line 41) [108] and PDGFβ-α-syn tg mice (line D) [109], have been previously described. The APP tg mice express mutated (London V717I and Swedish K670M/N671L) human APP751 under the control of the murine Thy1 promoter (Thy1-hAPP, line 41) [108]. This tg model was selected because mice produce high levels of Aβ_1–42_ and exhibit performance deficits in the water maze, synaptic damage, and plaque formation at an early age (beginning at 3 months) [108], [110]. Heterozygous APP and −α-syn tg mice were crossed as described before [31] to obtain double tg animals. Transgenic lines were maintained by crossing heterozygous tg mice with non-tg C57BL/6×DBA/2 F1 breeders. All mice were heterozygous with respect to the transgene.

### Immunoblot analysis

To analyze the distribution and levels of α-syn and Aβ in the brains of patients with DLB and in tg mice, briefly as previously described, samples from the frontal cortex were homogenized and fractioned into cytosolic and membrane fractions by ultracentrifugation. Approximately 20 µg of protein per lane were loaded into 4–12% Bis-Tris gels with 3-{N-morpholino] propanesulfonic acid (MOPS)/SDS buffer and blotted onto polyvinylidene fluoride (PVDF) membranes. Blots were incubated with antibodies against Aβ (6E10, 1∶1000, Signet) and α-syn (1∶1000, Chemicon, Temecula, CA), followed by secondary antibodies tagged with horseradish peroxidase (HRP, 1∶5000, Santa Cruz Biotechnology, Inc., Santa Cruz, CA) and visualized by enhanced chemiluminescence and analyzed with a Versadoc XL imaging apparatus (BioRad, Hercules, CA). Analysis of actin levels was used as a loading control.

To determine the effects of Aβ on α-syn aggregation, recombinant α-syn (1 µM, Calbiochem, San Diego, CA) was incubated in the presence or absence of freshly-solubilized or aggregated Aβ_1–42_ (10–20 µM, American Peptide, Sunnyvale, CA) at 37°C for 16 h {Hashimoto, 1998 #2038}. Additional experiments were performed by incubating recombinant α-syn (10 µM, Calbiochem) with wildtype (1–17) or mutated Aβ peptides (PHE4SER, GLU11ARG, VAL12SER, LYS16ASP) (custom-made by Invitrogen, Carlsbad, CA) at 20 µM followed by immunoblot analysis with the mouse monoclonal antibody against α-syn (LB509, 1∶1000, Zymed Laboratories, San Francisco, CA) or Aβ (6E10) as previously described [111] and analyzed in the VersaDoc imaging system using the Quantity One software (BioRad, Hercules, CA).

RETRACTED

### Lipid monolayer assay

A synthetic lipid monolayer was generated as described by Ford, M. *et al.* [112]. Briefly, cholesterol, phosphatidylethanolamine and phosphatidylcholine (all from Sigma) were dissolved in chloroform at a concentration of 10 mg/mL. Phosphatidylinositol-4,5-biphosphate (also from Sigma) was dissolved at 1 mg/mL in 3∶1 chloroform∶methanol. Lipid stocks were stored at −80°C. A monolayer of lipid containing 10% cholesterol, 40% phosphatidylethanolamine, 40% phosphatidylcholine and 10% phosphatidylinositol-4,5-biphosphate (at a final concentration of 0.1 mg/mL) in a 19∶1 mixture of chloroform methanol was formed on the surface of a 100 mM Tris/HCl/1 mM dithiothreitol buffer droplet in a Teflon block (kind gift of Dr. Harvey McMahon). After 1 hr incubation at room temperature, a carbon-coated gold electron microscopy grid [gold/mesh 100 formvar carbon film (EMS, Hatfield, PA)] was placed onto the monolayer and 10 µM recombinant α-syn (Calbiochem); 10 µM Aβ_1–42_ (American Peptide) alone or an equimolar mixture of both proteins were introduced into the buffer. After 6 hrs incubation at room temperature in a humid chamber, the grid was removed and stained with uranyl acetate (1% uranyl acetate) for 5 min and 2% bismuth subnitrate for 3 min, and analyzed by electron microscopy.

### Electron microscopy studies of α-syn and Aβ aggregates

To investigate the ultrastructural characteristics of the Aβ/α-syn aggregates, 1 µl aliquots of α-syn alone or in combination with Aβ prepared under identical conditions as for immunoblotting were pipetted onto formvar coated grids, followed by 2% uranyl acetate staining. Grids were analyzed with a Zeiss OM 10 electron microscope as previously described [111]. To estimate the number of ring-like structures formed, 10 random fields were analyzed at 50,000× magnification per condition. For each condition, three different grids were analyzed. The average number of ring-like structures was analyzed with digitized images using the ImageJ program (NIH). In each case a minimum of 100 rings was included for analysis. Results were expressed as mean per 1000 nm^2^.

### Preparation and electrophysiological analysis of cells expressing α-syn and treated with Aβ

HEK293T cells were grown on 25-mm coverslips at 50% confluence and were incubated with lentiviruses expressing α-syn or GFP (each at 1.0×10^7^ TU) in 10% fetal calf serum (FCS) for 24 h at 37°C, 5% CO_2_. Lentiviruses were prepared as previously described [113]. The cells were then washed with phosphate-buffered saline (PBS) and incubated in DMEM with 10% FCS for an additional 4 days. The efficiency of transduction of lenti-GFP was more than 90%. For electrophysiological measurements, whole-cell cation currents were recorded with an Axopatch-1D amplifier and a DigiData 1200 interface (Axon Instruments, Sunnyvale, CA) using patch-clamp techniques. Patch pipettes (2–3 MΩ) were fabricated on a Sutter electrode puller using borosilicate glass tubes and fire polished on a Narishige microforge. Command voltage protocols and data acquisition were performed using pCLAMP-8 software (Axon Instruments). All experiments were performed at room temperature (22–24°C). The ionic composition of the external solution was (in mM): NaCl 145, KCl 5, MgCl_2_ 1, CaCl_2_ 2, glucose 10, and HEPES 10 (pH = 7.4). During patch-clamp recording, tetrodotoxin (0.1 µM) and CdCl_2_ (0.1 mM) were added to the external solution to block voltage-dependent Na^+^ and Ca^2+^ channels. The ionic composition of the pipette solution was (in mM): CsCl 150 and HEPES 10 (pH = 7.2). The current-voltage (I–V) relationship was determined by a step voltage protocol of 50 ms duration. The cell was held at −50 mV and stepped to levels between −80 mV and +80 mV in 20-mV increments.

RETRACTED

For verification of α-syn expression after lentivirus infection, transduced cells were harvested in lysis buffer and analyzed by immunoblot with an antibody against α-syn (1∶1000, Chemicon). For immunocytochemistry, cells were cultured on cover slips until 50% confluence and treated as described above, fixed in 4% paraformaldehyde for 20 min, and blocked overnight at 4°C in 10% FCS and 5% bovine serum albumin. Cells on coverslips were then incubated overnight at 4°C with the antibody against α-syn (1∶2500, Chemicon). The following day, the antibody was detected with the Tyramide Signal Amplification-Direct (Red) system (NEN Life Sciences). Coverslips were air dried overnight, mounted on slides with anti-fading media (Vectashield, Vector Laboratories, Burlingame, CA), and imaged with the laser scanning confocal microscope (LSCM, MRC1024, BioRad). Co-localization with GFP was visualized with the endogenous green fluorescence of GFP.

### Calcium mobilization assay

Assessment of calcium influx was carried out using a modified protocol of the FLIPR 4 calcium assay (Molecular Devices, Sunnyvale, CA). Briefly, HEK293T cells were infected with lentiviral constructs harboring human wt α-syn (lenti-α-syn) or no extra DNA (lenti-empty). Cells infected at a MOI of 30 were cultured in DMEM medium (Mediatech, Manassas, VA) containing 10% FBS and penicillin/streptomycin. Cultures were maintained in an incubator at 37° C, in an atmosphere of 95% air and 5% CO_2_. Two days after infection, cells were plated at a density of 30,000 cells/well on Costar 96 well-black plates with flat clear bottom (Corning, Corning, NY). Cells were treated for 24 hr with control vehicle or freshly solubilized Aβ_1–42_ (10 µM American Peptide). After treatment, media was replaced by 100 µl of HBSS buffer and 100 µl of calcium dye was added to each well. Cells were kept in the incubator at 37°C for 1 hr before measuring fluorescence with excitation/emission filter at 470–495/515–575 nm on a DTX 880 Multimode Detector (Beckman Coulter, Fullerton, CA). As a positive control of calcium influx, 0.6 µg of ionomycin (Sigma, St. Louis, MO) was added to the indicated wells.

RETRACTED

### Statistical analysis

The data are expressed as mean values±standard error of the mean (SEM). Statistical analysis was performed using one-way analysis of variance (ANOVA) followed by post hoc Dunnett's or Tukey-Kramer tests (Prism Graph Pad Software, San Diego, CA, USA). The significance level was set at p<0.05.

## Supporting Information

Figure S1 Molecular dynamics simulations of Aβ conformers at various time points. (A) Initial conformer; (B) 0.5 ns conformer; (C) 1.0 ns conformer; (D) 1.5 ns conformer; (E) 2.0 ns conformer; (F) 2.5 ns conformer; (G) 3.0 ns conformer; and (H) superimposed image showing all conformers in a composite image.
(0.69 MB TIF)

Figure S2 Molecular dynamics simulations showing the changes in Aβ secondary structure over time. The first time zero line shows the amino acid sequence of Aβ1–42, and the remaining lines depict the secondary structural characteristics.
(0.86 MB TIF)

Figure S3 Molecular dynamics simulations of α-syn multimers with Aβ monomers and dimers. The 4 ns α-syn dimer and the 2 ns Aβ conformer were used for modeling all complexes. (A) Structural organization of one α-syn dimer complexed with one Aβ monomer. (B) Structural organization of one α-syn trimer complexed with two Aβ monomers. (C) Structural organization of one α-syn pentamer complexed with two Aβ monomers. (D) Structural organization of one α-syn dimer complexed with one Aβ dimer. (E) Structural organization of one α-syn trimer complexed with one Aβ dimer. (F) Structural organization of one α-syn pentamer complexed with one Aβ dimer.
(1.04 MB TIF)

Figure S4 Increased levels of α-syn multimers in the presence of Aβ under in vitro aggregating conditions. Freshly-solubilized recombinant α-syn (10 µM) and freshly-solubilized Aβ (5–20 µM) were incubated together at the indicated ratios for 24 hrs and analyzed by immunoblot. (A) Incubation of α-syn with Aβ promotes the formation of a 170-kDa oligomer of α-syn. (B) Semi-quantitative analysis of α-syn multimer levels showing increasing levels of α-syn dodecamer with increasing Aβ concentration. In cases where no α-syn recombinant protein was included (negative control), no immunoreactivity was detected with the antibody against α-syn.
(0.28 MB TIF)

Figure S5 Analysis of intracellular calcium levels in cells expressing α-syn and treated with Aβ. 293T cells were infected with lenti-vector or lenti-α-syn for two days and treated with 10 µM freshly-solubilized Aβ1–42 for 24 hrs, followed by treatment with calcium dye and analyzed by fluorescence microscopy and with a spectrophotomer. (A) Minimal calcium dye uptake in cells infected with vector control. (B, C) Moderate calcium dye uptake in cells expressing α-syn (B) or exposed to Aβ (C). (D) High calcium dye uptake in cells expressing α-syn and treated with Aβ. (E) Levels of calcium dye uptake, expressed in terms of relative fluorescence units (RFU). *P<0.05 compared to vector-infected controls (by one-way ANOVA with post-hoc Dunnett's test); **P<0.05 compared to cells expressing α-syn or treated with Aβ alone (by one-way ANOVA with post-hoc Tukey-Kramer test).
(0.38 MB TIF)
